# Osimertinib Improves Overall Survival in Patients with Leptomeningeal Metastases Associated with *EGFR*-Mutated Non-Small-Cell Lung Cancer Regardless of Cerebrospinal Fluid T790M Mutational Status

This article has been retracted.

**DOI:** 10.1155/2021/6968194

**Published:** 2021-08-19

**Authors:** Milan Zhang, Weifeng Ma, Huiqin Liu, Yushu Jiang, Lingzhi Qin, Wei Li, Jiewen Zhang

**Affiliations:** Department of Neurology, People's Hospital of Zhengzhou University, Henan Provincial People's Hospital, Weiwu Rd 7, Zhengzhou 450003, Henan, China

## Abstract

Osimertinib has demonstrated promising efficacy against leptomeningeal metastasis (LM) associated with T790M-positive non-small-cell lung cancer (NSCLC). However, the effect of cerebrospinal fluid's (CSF's) epidermal growth factor receptor (*EGFR*) T790M mutation on osimertinib efficacy remains unclear.Seventy-eight patients were studied with *EGFR*-mutated NSCLC and LM. Case data were collected and *EGFR* mutation status of circulating cell-free DNA from paired CSF, and plasma of 23 patients with LM was detected using droplet digital PCR. The median overall survival (mOS) was 8.08 months (95% CI: 6.07–10.09) in the study. Forty-four osimertinib-treated patients had an improved mOS of 13.15 (95% CI: 5.74–20.57) and a median progression-free survival (PFS) of 9.50 months (95% CI: 6.77–12.23) when compared with patients treated with first- or second-generation *EGFR*-TKI (mOS = 3.00 months (95% CI: 1.32–4.68) and median PFS = 1.50 months (95% CI: 0.00–3.14)). In the osimertinib group, mOS values for CSF with and without T790M mutation were 22.15 months (95% CI: 9.44–34.87) and 13.39 months (95% CI: 7.01–19.76), respectively, with no statistical differences. Regardless of the CSF T790M mutation status, osimertinib demonstrated significant efficacy against LM associated with NSCLC.

## 1. Introduction

Leptomeningeal metastasis (LM) is defined as the spread of malignant cells within the leptomeninges and subarachnoid space, resulting in a devastating prognosis with limited treatment options [1]. Non-small-cell lung cancer (NSCLC) is the most common primary tumor of LM, and epidermal growth factor receptor (*EGFR*) is the most important driver gene in NSCLC. *EGFR* mutations occur in 10–20% of Caucasian patients with NSCLC but in 40–60% of Asian patients [2]. The detection rate of LM in patients with NSCLC has been estimated to be 3–4% but 9–16% in patients with lung adenocarcinoma harboring *EGFR* mutations [3, 4]. This difference may partly be because of improved overall survival (OS) conferred by *EGFR* tyrosine kinase inhibitor (*EGFR-*TKI) treatments [4].

*EGFR* mutation status is a critical prognostic factor in the treatment of NSCLC with LM. A secondary *EGFR* test is often required to determine the status of T790M drug-resistant mutation. However, it is difficult to obtain a second tumor tissue from most patients. Circulating cell-free DNAs (cfDNAs) are extracellular nucleic acids released by tumor cells that can be useful biomarkers for early diagnosis and prognosis [5]. However, because of the blood-brain barrier, the role of plasma cfDNA in the diagnosis of metastatic brain cancer is very limited. Nevertheless, the enrichment of cerebrospinal fluid (CSF) with intracranial tumor cfDNA has become increasingly emphasized in intracranial tumor fluid biopsies [6, 7].

LM is often associated with an extremely poor prognosis, with a median OS (mOS) of 3–10 months after diagnosis [8]. Currently, the options for systemic therapy for LM are limited; additionally, the efficacy of first-generation (erlotinib and gefitinib) and second-generation (afatinib) *EGFR*-TKIs remains dismal [9–13]. Although second-generation *EGFR-*TKIs, such as afatinib, could partially penetrate the blood–brain barrier, they exhibit no obvious advantage as a treatment for LM [13].

Osimertinib is an irreversible third-generation *EGFR*-TKI that selectively inhibits *EGFR* and *EGFR* T790M mutations. It is highly effective in both untreated and previously treated patients with *EGFR*-mutated NSCLC by prolonging OS and progression-free survival (PFS) [14–16]. According to the BLOOM study, high-dose osimertinib (160 mg daily) resulted in a mOS of 11.0 months for pretreated patients with LM associated with *EGFR*-mutated positive NSCLC [15]. In contrast, the AURA study reported improved survival, with a mOS of 18.8 months in the osimertinib treatment cohort for patients harboring the *EGFR* T790M mutation [16].

Few studies have focused on the relationship between CSF *EGFR* T790M mutation status and osimertinib efficacy in patients with NSCLC [17, 18]. In this study, we aimed to develop a droplet digital PCR (ddPCR) method to detect plasma and CSF cfDNA, to compare the clinical efficacy of osimertinib with first- or second-generation *EGFR-*TKIs and evaluate the factors influencing osimertinib efficacy.

## 2. Materials and Methods

### 2.1. Patients

This retrospective study involved patients with *EGFR*-mutated NSCLC and LM at the People's Hospital of Zhengzhou University, recruited from January 1, 2014, to December 31, 2020. Inclusion criteria were: (1) space-occupying lesions of the lungs detected using computed tomography (CT) or whole-body positron emission tomography/computed tomography (PET/CT) and confirmed as NSCLC using histological biopsy, (2) symptoms and signs of the central nervous system metastases, (3) typical leptomeningeal enhancement on magnetic resonance imaging (MRI), and (4) cytologic identification of malignant cells within the CSF. All patients were scored using the Eastern Cooperative Oncology Group performance status (ECOG PS), CT, or PET/CT. In addition, the patient's histology, metastasis site, imaging, CSF parameters, and molecular profiling were collected. And no patients had complicated organ failure, infection in the central nervous system, and diseases of the autoimmune system or hematological system.

Among the 78 patients with *EGFR*-mutated NSCLC and LM, 34 patients were treated with first- or second-generation EGFR-TKIs treatment, and 44 patients (41.5%, including 28 patients with T790M mutation and 16 patients without T790M mutation) were treated with osimertinib (Figure 1).

### 2.2. EGFR Mutations

*EGFR* mutations were initially detected via tissue biopsy using amplification refractory mutation system polymerase chain reaction (ARMS-PCR) analysis or next-generation sequencing.

Secondary T790M mutation analysis was performed using one of the following samples: biopsied tumor tissues, plasma, or CSF samples. Approximately 10 mL of whole blood and 10 mL of CSF (EDTA as the anticoagulant) were collected for the purpose of cfDNA extraction. The retrieved CSF was used for analysis within 4 h of the lumbar puncture procedure. Plasma and CSF were centrifuged at 1,600 × g and 10,000 × g, respectively, for 10 min at room temperature. CfDNA was extracted using the QiAamp circulating nuclear acid kit (Qiagen, Hilden, Germany). Droplet digital PCR (ddPCR) was used to detect cfDNA using the Sysmex OncoBeam *EGFR* kit (SYSMEX, Japan). All protocols of analysis were carried out in strict accordance with the manufacturer's instructions.

### 2.3. Follow-Up

OS for LM was defined as the time from LM diagnosis to death. PFS was calculated from the onset of *EGFR*-TKI treatment to tumor progression. The cutoff date was December 31, 2020.

### 2.4. Statistical Analyses

Statistical analyses were performed using SPSS software (IBM statistics, version 22). Chi-square univariate analysis was used for continuous variables, and a non-parametric test was used for non-normal distribution variables. Kaplan–Meier estimation and log rank *p* values were used for survival analysis at 95% confidence intervals (95% CI). Cox regression analysis was performed to estimate hazard ratios (HRs) and 95% CIs for OS. Statistical significance was set at *p* < 0.05.

## 3. Results

### 3.1. Baseline Features

As shown in Table 1, a total of 78 *EGFR*-mutated NSCLC and LM were included. The median age was 61 years (range: 28–78), and 74.4% (58/78) were non-smokers. The ECOG PS scores at the time of LM diagnosis were: <1 in 23 (29.5%), 2–3 in 43 (55.1%), and 4 in 12 patients (15.4%). Twenty-five patients with NSCLC also presented with LM at initial diagnosis. The median time from NSCLC to LM diagnosis of the remaining 53 patients was 21 months (95% CI: 12.0–24.5). Statistically significant differences were not observed in age, sex, smoking status, histology, initial ECOG PS scores, and *EGFR* mutations.

### 3.2. EGFR Mutation Analysis

Among the 78 patients, 66 (84.6%) of them underwent secondary *EGFR* T790M mutation analysis. Of these samples, *EGFR* T790M mutation was identified in 28 cases.

Plasma and CSF were used to detect the *EGFR* gene of cfDNA in 23 patients simultaneously, and T790M mutation was detected in 8 patients (Supplementary Table 1). The detection rates of *EGFR* mutations in plasma and CSF samples were 56.5% (13/23) and 60.9% (14/23), respectively, but without any statistically significant difference (*p*=0.765).

### 3.3. Treatment of LM

Prior to LM diagnosis, 53 patients had undergone at least 1 treatment with early generation *EGFR*-TKI: 24 (45.3%) of them received gefitinib, 11/53 (20.8%) received erlotinib, 7/53 (13.2%) received icotinib, 5/53 (9.4%) received afatinib and gefitinib, and 6/53 (11.3%) received osimertinib. Moreover, 35/53 (66.0%) patients received cytotoxic chemotherapy, and 11/53 (20.8%) had undergone whole-brain radiation therapy (WBRT) for brain metastasis prior to LM (Table 2).

Forty-four patients (including 28 patients with T790M mutation and 16 patients without T790M mutation) were treated with osimertinib at the time of LM diagnosis. The median duration of osimertinib treatment was 7.0 months (95% CI: 4.0–9.0). Table 2 summarizes the osimertinib treatment line, dosage, and supplementary treatments.

Thirty-four patients received first- or second-generation TKI treatment without osimertinib. Eighteen (52.9%) of them received gefitinib; 10 (29.4%) received erlotinib; 3 (8.8%) received icotinib; and 1 (2.9%) received afatinib and gefitinib. Twelve patients (35.7%) received cytotoxic chemotherapy; 4 (12.9%) received WBRT; 2 (6.5%) underwent IT chemotherapy; and 3 (9.7%) had VPS insertion (Table 2).

### 3.4. Clinical Responses and OS

At the end of follow-up, 58 patients died from the disease, 15 were still alive, and 5 were lost to follow-up (6.4%). The 1-year OS rate in the study was 32.7% (19/73), with a mOS of 8.08 months (95% CI: 6.07–10.09; Figure 2(a)).

Among the 44 patients who received osimertinib treatment, 39 (88.6%) had positive clinical responses. Twenty-eight patients died, and 14 were still alive at the time of follow-up, with a mOS of 13.15 months (95% CI: 5.74–20.57). The 1-year OS rate was 53%. Among the patients who were treated with first- or second-generation *EGFR*-TKI, 30 had died, and only 1 was alive. The mOS was only 3.00 months (95% CI: 1.32–4.68), with a 1-year OS rate of 12.9%, which was shorter than that of patients treated with osimertinib (HR: 0.58 (95% CI: 0.44–0.77) and *p* ≤ 0.001; Figure 2(b)).

Compared to the group treated with osimertinib, PFS of the group treated without osimertinib also was significantly shorter (PFS: 1.50 months (95% CI: 0.00–3.14) and HR: 0.57 month (95% CI: 0.44–0.75); Figure 2(c)).

Furthermore, we further divided the group treated with osimertinib into two subgroups according to T790M mutational status. The mOS for patients with and without T790M mutational status was 15.92 months (95% CI: 7.70–24.14) and 9.00 months (95% CI: 5.50–12.50), respectively, but without any significant difference (*p*=0.564). Regardless of T790M status, the survival benefit of the osimertinib treatment group was better than that of the first- or second-generation *EGFR*-TKI treatment group (mOS = 3.00 months (95% CI: 1.32–4.68) and HR: 0.56 (95% CI: 0.41–0.78); Figure 2(d)).

*EGFR* mutation in CSF cfDNA was detected in 23 patients of the osimertinib treatment group. Seven patients with T790M mutation in CSF had a mOS of 22.15 months (95% CI: 9.44–34.87), whereas 16 patients without T790M mutation had a mOS of 13.39 months (95% CI: 7.01–19.76). No statistical difference was found according to Kaplan–Meier survival analysis (Figure 2(e)).

Thirty-one patients were administered 80 mg osimertinib daily, whereas 13 patients were administered 160 mg daily; the mOS of patients receiving the 2 different dosages was 10.0 months (95% CI: 4.48–15.52) and 13.39 months (95% CI: 3.59–23.18), respectively. However, survival analysis revealed no significant differences between the two groups (*p*=0.416; Figure 2(f)).

### 3.5. Univariate and Multivariate Analyses

Based on univariate and multivariate analyses, a higher ECOG PS score was associated with a worse prognosis (univariate HR: 3.95 (95% CI: 2.19–7.10), *p*=0.001 and multivariate HR: 3.22 (95% CI: 1.74–5.95), *p*=0.021). Osimertinib treatment was identified as a significant independent favorable prognostic factor in patients with NSCLC and LM (univariate HR: 0.59 (95% CI: 0.45–0.78), *p*=0.000 and multivariate HR: 0.65 (95% CI: 0.49–0.87), *p*=0.004). Univariate analysis revealed a statistically significant correlation between WBRT and prognosis (0.45 (95% CI: 0.23–0.96), *p*=0.038). However, no significant associations were observed with concurrent brain metastases, initial *EGFR* and *EGFR* T790M mutations, CSF pressure, protein and glucose levels, and systemic and intrathecal cytotoxic chemotherapy (Table 3).

## 4. Discussion

The treatment of lung cancer has gradually evolved from traditional therapies to gene-oriented personalized treatments. The first- and second-generation *EGFR*-TKI drugs have resulted in significant survival benefits and improved quality of life for patients with *EGFR* mutations. Third-generation *EGFR*-TKIs, such as osimertinib, have also been found to extend the survival of patients with T790M mutation by more than 10 months [16].

Our study found that osimertinib is a clinically effective standard regimen in patients with LM associated with *EGFR* + NSCLC, regardless of T790M mutation that confers drug resistance, with a median LM PFS of 9.50 months and a mOS of 13.15 months. Patients treated with only first- or second-generation *EGFR*-TKI after LM diagnosis had a median PFS of 1.50 months and a mOS of 3.00 months. Compared to first- or second-generation *EGFR*-TKIs, osimertinib showed a markedly improved survival benefit.

As mentioned, the efficacy of first-generation *EGFR*-TKIs for LM is limited because of the blood–brain barrier. The first- and second-generation *EGFR-*TKIs have low CSF penetration, with an average CSF penetration of 1–3% for gefitinib and 3–6% for erlotinib compared to only 1% for afatinib [9–13]. High-dose gefitinib (2-week dosage of 750–1,000 mg daily and then 2-week dosage of 500 mg daily) was ineffective to prolong patient survival [9]. Although erlotinib may have a better CSF cytological conversion rate than gefitinib, with an mOS of 3.4 months in the Phase II Study (LOGIK1101), the observed clinical response remains unsatisfactory [10].

Preclinical studies of osimertinib using mouse models of brain metastasis with 19 gene deletions (PC9) have demonstrated that a dose-dependent tumor reduction can be achieved [19]. The FLAURA study further confirmed the benefit of osimertinib as a first-line treatment drug for NSCLC with a median PFS of 18.9 months [14]. The AURA and AURA2 studies had verified the clinical efficacy of osimertinib in patients with BMs [20, 21]. The AURA3 study, which included 116 patients with central nervous system (CNS) metastases, confirmed that osimertinib exhibited a higher and more persistent response in patients with CNS metastases than the reported efficacy of the BLOOM study [16]. According to a BLOOM study, osimertinib 160 mg daily demonstrated systemic and CNS activities in patients with LM associated with *EGFR* mutation NSCLC [15]. Several small prospective and retrospective studies have suggested that the standard dosage of osimertinib (80 mg) may have similar efficacy to the 160 mg dosage and is an effective treatment option for refractory LM following classic *EGFR*-TKI therapy failure [22, 23]. Similar to previous studies, the present study found that high-dose (160 mg) osimertinib treatment for 13.39 months (95% CI: 3.59–23.18) did not improve OS compared to the standard dose (80 mg) for 10.0 months (95% CI: 4.48–15.52); however, we could not rule out the risk of bias due to the small number of patients in the 160 mg treatment group.

The excluded patients based on *EGFR* T790M screening failure in the BLOOM study might be a missed opportunity in revealing osimertinib activity in the CNS [15]. A recent retrospective study involving 351 patients with LM showed that mOS of patients with or without T790M mutation status under osimertinib treatment were 16.7 and 18.8 months, respectively [18]. Similarly, in this study, osimertinib treatment for patients with or without T790M mutational status yielded mOS of 15.92 and 9.00 months, respectively, and with no statistical difference. The efficacy of osimertinib in patients with LM due to *EGFR*-TKI-resistant NSCLC and without the T790M mutation should be further investigated.

Due to the blood–brain barrier, plasma cfDNA may not accurately reflect the actual state of mutations in intracranial tumors, whereas the rapid CSF circulation within the cerebral ventricle and spinal cord cavity indicates that CSF cfDNA may be a reliable biomarker for intracranial tumors. In patients with LM associated with metastasized lung carcinoma, the proportion of *EGFR* mutations detected using CSF cfDNA tended to be higher compared to plasma cfDNA [6]. A similar study involving 92 patients with NSCLC and LM of Han Chinese descendants revealed a 58% *EGFR* mutation rate based on CSF samples [7], which is consistent with the rate detected in the present study. CSF genotyping has been employed to predict the difference in the efficacy of osimertinib treatment in patients with LM due to NSCLC and reveal the underlying mechanism of drug resistance progression after osimertinib treatment [24]. However, in our study, no correlation was found between the status of CSF T790M mutation and the efficacy of osimertinib due to the small sample size. Therefore, next-generation sequencing (NGS) of CSF cfDNA will be a better assay to elucidate the relationship between gene mutations and osimertinib efficacy. The above findings can be used for comprehensive analysis *in vivo*, *in vitro*, and/or *in silico* along with other math tools and models, including meta-analysis [25, 26], research models [27, 28], network pharmacology [29], and molecular docking [30, 31].

This study had several limitations. Firstly, this was a retrospective study involving a small number of patients. All the patients included in our study were confirmed using cytological findings, whereas patients diagnosed via clinical examination and imaging were not included, which may have contributed to selection bias. Secondly, the ddPCR method for detecting plasma and CSF cfDNA had low sensitivity, which could have potentially resulted in a lower detection rate. Therefore, more sensitive cfDNA detection assays, such as NGS, will be employed for further verification analysis.

## 5. Conclusions

Case data were collected and *EGFR* mutation status of circulating cell-free DNA from paired CSF, and plasma of 23 patients with LM was detected using droplet digital PCR. The median overall survival (mOS) was 8.08 months (95% CI: 6.07–10.09) in the study. Forty-four osimertinib-treated patients had an improved mOS of 13.15 months (95% CI: 5.74–20.57) and a median progression-free survival (PFS) of 9.50 months (95% CI: 6.77–12.23) when compared with patients treated with first- or second-generation *EGFR*-TKI (mOS = 3.00 months (95% CI: 1.32–4.68) and median PFS = 1.50 months (95% CI: 0.00–3.14)). In the osimertinib group, mOS values for CSF with and without T790M mutation were 22.15 months (95% CI: 9.44–34.87) and 13.39 months (95% CI: 7.01–19.76), respectively, with no statistical differences. Regardless of the CSF T790M mutation status, osimertinib demonstrated significant efficacy against LM associated with NSCLC.

## Figures and Tables

**Figure 1:** Flow diagram of patient enrollment. NSCLC: non-small-cell lung cancer, LM: leptomeningeal metastasis, CSF: cerebrospinal fluid, *EGFR*: epidermal growth factor receptor, ALK: anaplastic lymphoma kinase, ROS1: ROS proto-oncogene 1, and TKI: tyrosine kinase inhibitor.

**Figure 2:** (a) Overall survival from LM diagnosis for the total population. (b) Kaplan–Meier curve of the OS of patients in the osimertinib and the first- or second-generation *EGFR*-TKI treatment groups. (c) Kaplan–Meier curve of the PFS of patients in osimertinib and the first- or-second generation *EGFR*-TKI treatment groups. (d) Kaplan–Meier estimates of OS according to osimertinib treatment and T790M mutation status. (e) Kaplan–Meier estimates of OS according to osimertinib treatment and CSF T790M mutation status. (f) Kaplan–Meier estimates of OS according to different osimertinib dosages. OS: overall survival, PFS: progression-free survival, TKI: tyrosine kinase inhibitor, CI: confidence interval, and HR: hazard ratio.

**Table 1:** Patient characteristics at the time of NSCLC diagnosis.

Patient characteristics	Osimertinib treated with T790M, *n* = 28 (%)	Osimertinib treated without T790M, *n* = 16 (%)	First-/second-generation *EGFR*-TKI, *n* = 34 (%)	*p* value
Age, year (range)	61 (32–78)	52 (28–68)	63 (41–73)	0.322
Median time to LM, months (95% CI)	15.0 (6.0–25.0)	12.5 (6.0–24.0)	3.5 (0.0–12.0)	0.566

Sex				0.408
Male	12 (42.9)	10 (62.5)	15 (44.1)	
Female	16 (57.1)	6 (37.5)	19 (55.9)	

Smoking status				0.083
Current or former	8 (28.6)	7 (43.8)	5 (14.7)	
Never	20 (71.4)	9 (56.2)	29 (85.3)	

Number of metastatic sites, *n* (%)				0.567
≤2	6 (24.0)	5 (35.7)	11 (36.7)	
≥3	19 (76.0)	9 (64.3)	19 (63.3)	

Histology				0.415
Adenocarcinoma	27 (96.4)	16 (100.0)	34 (100.0)	
Adenosquamous carcinoma	1 (3.6)	0	0	

ECOG PS score at LM Dx				0.097
0–1	9 (32.1)	6 (37.5)	8 (23.5)	
2–3	18 (64.3)	7 (43.8)	18 (52.9)	
4	1 (3.6)	3 (18.8)	8 (23.5)	

*EGFR* mutation				0.707
Exon 19	14 (50.0)	11 (68.8)	17 (50.0)	
Exon 21	12 (42.9)	4 (25.0)	17 (50.0)	
Exon 18	2 (7.1)	1 (6.2)	0	

*Note.* NSCLC: non-small-cell lung cancer, ECOG PS: Eastern Cooperative Oncology Group performance status, and *EGFR*: epidermal growth factor receptor.

**Table 2:** Osimertinib and supplementary treatments for LM.

Characteristics	Osimertinib with T790M, *n* = 28 (%)	Osimertinib without T790M, *n* = 16 (%)	First-/second-generation *EGFR*-TKI, *n* = 34 (%)
Treatments prior to LM			
Gefitinib only	5 (17.9)	8 (50.0)	11 (32.4)
Erlotinib only	2 (7.1)	2 (12.5)	7 (20.6)
Icotinib only	6 (21.4)	1 (6.3)	0 (0)
Afatinib and gefitinib	3 (10.7)	2 (12.5)	0 (0)
Osimertinib	5 (17.9)	1 (6.3)	0 (0)
Cytotoxic chemotherapy	15 (53.6)	11 (68.8)	9 (26.5)
WBRT	3 (10.7)	3 (1 8.8)	5 (14.7)
Median duration of osimertinib treatment, months (95% CI)	7.0 (4.0–10.0)	7.0 (1.5–10.0)	—

Osimertinib treatment line			
1^st^ line	0	4 (25.0)	—
2^nd^ line	17 (60.7)	8 (50.0)	—
3^rd^ line	11 (39.3)	4 (25.0)	—

Osimertinib dosage			
80 mg/day	19 (67.9)	12 (75.0)	—
160 mg/day	9 (32.1)	4 (25.0)	—

Supplementary treatments			
Cytotoxic chemotherapy	17 (60.7)	11 (68.8)	12 (38.7)
WBRT	5 (17.9)	3 (18.8)	4 (12.9)
IT chemotherapy	7 (25.0)	5 (31.3)	2 (6.5)
VPS	3 (10.7)	4 (25.0)	3 (9.7)

*Note.* LM: Leptomeningeal metastasis, WBRT: whole-brain radiation, IT: intrathecal, and VPS: ventriculoperitoneal shunt.

**Table 3:** Univariate and multivariate analyses of OS from LM diagnosis.

Variables	*n*	Univariate analysis		Multivariate analysis	
		HR (95% CI)	*p* value	HR (95% CI)	*p* value
Age, year					
≤60	38	1.00	—	—	—
>60	40	0.85 (0.50–1.42)	0.525	—	—

Sex					
Male	37	1.00	—	—	—
Female	41	0.95 (0.56–1.61)	0.859	—	—

Smoking					
No	58	1.00	—	—	—
Yes	20	1.58 (0.85–2.96)	0.147	—	—

ECOG PS					
0–2	49	1.00	—	1.00	—
≥3	29	3.95 (2.19–7.10)	≤0.001	3.22 (1.74–5.95)	≤0.001

Concurrent BM					
No	38	1.00	—	—	—
Yes	33	1.07 (0.62–1.85)	0.807	—	—

Initial *EGFR* mutation					
19DEL	42	1.00	—	—	—
21L8585R	33	1.06 (0.63–1.80)	0.823	—	—
Other	3	1.16 (0.56–2.40)	0.685	—	—

*EGFR* T790M mutation					
Present	28	1.00	—	—	—
Absent	38	1.60 (0.89–2.90)	0.118	—	—

CSF pressure, mmH_2_O					
≤180	25	1.00	—	—	—
>180	49	0.94 (0.53–1.65)	0.828	—	—

CSF protein, mg/dl					
≤50	23	1.00	—	—	—
>50	44	0.99 (0.53–1.87)	0.987	—	—

CSF glucose, mmol/L					
≥2.5	25	1.00	—	—	—
<2.5	43	1.08 (0.60–1.94)	0.808	—	—

Cytotoxic chemotherapy					
No	35	1.00	—	—	—
Yes	40	0.87 (0.50–1.51)	0.625	—	—

IT chemotherapy					
No	59	1.00	—	—	—
Yes	14	0.63 (0.30–1.34)	0.227	—	—

WBRT					
No	63	1.00	—	1.00	—
Yes	13	0.45 (0.23–0.96)	0.038	0.77 (0.34–1.75)	0.539

VPS insertion					
No	66	1.00	—	—	—
Yes	10	0.79 (0.39–1.58)	0.498	—	—

Osimertinib treatment					
No	34	1.00	—	1.00	—
Yes	44	0.59 (0.45–0.78)	≤0.001	0.65 (0.49–0.87)	0.004

*Note.* HR: hazard ratio, CI: confidence interval, ECOG PS: Eastern Cooperative Oncology Group performance status, BM: brain metastases, IT: intrathecal, WBRT: whole-brain radiation therapy, and VPS: ventriculoperitoneal shunt.

## Data Availability

The data used to support the findings of this study are included within the article and the supplementary information file.

## Supplementary Materials

Supplementary Materials Supplementary Table 1: detection of T790M in paired *EGFR* mutations in plasma and CSF of patients with NSCLC and LM. .
